The article "Pattern and Determinants of Antiretroviral Drug Adherence among Nigerian Pregnant Women" was published in 2012. Journal: J Pregnancy.

# Pattern and Determinants of Antiretroviral Drug Adherence among Nigerian Pregnant Women

**DOI:** 10.1155/2012/851810

**Published:** 2012-02-23

**Authors:** S. O. Ekama, E. C. Herbertson, E. J. Addeh, C. V. Gab-Okafor, D. I. Onwujekwe, F. Tayo, O. C. Ezechi

**Affiliations:** ^1^Clinical Sciences Division, Nigerian Institute of Medical Research, P.M.B 2013, Yaba, Lagos, Nigeria; ^2^Department of Clinical and Biopharmacy, Faculty of Pharmacy, University of Lagos, P.M.B 12003, Surulere, Lagos, Nigeria

## Abstract

*Background*. The need for a high level of adherence to antiretroviral drugs has remained a major hurdle to achieving maximal benefit from its use in pregnancy. This study was designed to determine the level of adherence and identify factors that influence adherence during pregnancy. *Method*. This is a cross-sectional study utilizing a semistructured questionnaire. Bivariate and multiple logistic regression models were used to determine factors independently associated with good drug adherence during pregnancy. *Result*. 137 (80.6%) of the interviewed 170 women achieved adherence level of ≥95% using 3 day recall. The desire to protect the unborn child was the greatest motivation (51.8%) for good adherence. Fear of being identified as HIV positive (63.6%) was the most common reason for nonadherence. Marital status, disclosure of HIV status, good knowledge of ART, and having a treatment supporter were found to be significantly associated with good adherence at bivariate analysis. However, after controlling for confounders, only HIV status disclosure and having a treatment partner retained their association with good adherence. *Conclusion*. Disclosure of HIV status and having treatment support are associated with good adherence. Maternal desire to protect the child was the greatest motivator for adherence.

## 1. Introduction

The introduction of highly active antiretroviral therapy (HAART) has not only improved longevity in HIV-infected individuals but in addition has had a significant impact on the rate of mother-to-child transmission of HIV infection (MTCT) [1]. Mother-to-child transmission is one of the modes of HIV transmission. Vaginal delivery contributes 60–70% of MTCT, breastfeeding contributes 20–30%, while *in-utero* infection could occur in less than 10% of MTCT [2]. Without preventive intervention, about 25–40% of infants born to HIV-positive mothers will contract the virus [2]. Following introduction of HAART, the rates of mother-to-child transmission of HIV infection has practically crashed to less than 2% [3, 4]. However, the success of HAART, like any medication, is dependent on both the intrinsic properties of the drugs and the individual's ability to take the medication as prescribed [5]. This is particularly true in the prevention of mother-to-child transmission, where the consequence of failing to achieve viral suppression is the transmission of the virus to the baby [5]. Adequate adherence to the prescribed antiretroviral medications is essential to achieving maximal viral suppression necessary to prevent MTCT [4].

The article "Pattern and Determinants of Antiretroviral Drug Adherence among Nigerian Pregnant Women" was published in 2012. Journal: J Pregnancy.

Adherence rates exceeding 95% are necessary, in order to maximize the benefits of antiretroviral therapy. Higher levels of drug adherence are associated with improved virological, immunological, and clinical outcome [6].

Poor adherence to antiretroviral drugs during pregnancy can lead to suboptimal viral suppression, development of viral resistance, higher risk of mother-to-child transmission, and mother-to-child transmission of resistant HIV strains [5].

Interrupting medication permits the virus to resume rapid replication and as many as 10^10^ viral particles will be produced per day [7].

This allows resistant mutant strains to be generated which are no longer responsive to available antiretroviral drugs, posing a public health danger [7].

Adherence to antiretroviral drugs poses unique challenges to HIV infected persons particularly in pregnant women [7]. Improving adherence among pregnant women therefore requires knowledge of the factors that influence adherence.

Several methods have been used to measure adherence, but no gold standard has been established [8]. Each of these methods has its respective strengths and weaknesses. Available methods include pill counts, self-report, prescription refills, medication event monitoring system (MEMS), biological markers, and assays [4, 9].

Though several studies in Nigeria have evaluated the factors associated with nonadherence to antiretroviral therapy among HIV-positive adults [10–12], only one from literature search studied antiretroviral adherence issues in HIV-positive pregnant women [4].

They deduced from their study that the determinants of nonadherence to antiretroviral drugs in HIV-positive pregnant women were low level of education, nondisclosure of HIV status, and longer duration of therapy [4].

Good adherence is imperative for the success of PMTCT. This study, therefore, seeks to find out if there is good adherence to antiretroviral drugs among HIV-positive pregnant women.

 The main objective of this study is to determine the level and factors that influence adherence to antiretroviral drugs among HIV-positive pregnant women accessing PMTCT services in Lagos Nigeria.

**Research Questions**

1. What is the level of adherence to antiretroviral drugs among pregnant women?
2. What are the barriers to adherence in pregnancy?
3. What factors facilitate adherence among pregnant women?

The article "Pattern and Determinants of Antiretroviral Drug Adherence among Nigerian Pregnant Women" was published in 2012. Journal: J Pregnancy.

## 2. Method

### 2.1. Study Setting

The study was conducted at the HIV treatment Centre of the Nigerian Institute of Medical Research (NIMR), Lagos, a Federal Government of Nigeria Comprehensive HIV Care and Treatment Centre. NIMR is supported by AIDS Prevention Initiative in Nigeria (APIN) through the United States president's emergency fund for AIDS relief (PEPFAR), funding since 2004. The Centre provides an outpatient Prevention of Mother-To-Child-Transmission of HIV Infection (PMTCT) services, in addition to adult and pediatric HIV services. Pregnant women who tested positive to HIV are referred from the NIMR HIV counseling and testing centre or other public and private health institutions to the PMTCT clinic which takes place once a week, on Wednesdays. Intrapartum care is provided for these women in collaboration with some hospitals within Lagos metropolis which include Lagos University Teaching Hospital Idi Araba, Lagos State University Teaching Hospital Ikeja, General Hospital Surulere, General Hospital Apapa, General Hospital Ikorodu, Havana Specialist Hospital Surulere, and Rao Specialist Hospital Surulere. Antenatal, postnatal, and infant post exposure prophylaxes are provided by NIMR. Health workers from the collaborating centres have been trained on intrapartum care of HIV-positive mothers both by NIMR and the national HIV programme. Each woman on the PMTCT programme is referred to any of the collaborating centres, close to their place of residence at 36 weeks or as soon as possible for late booking. The referral note usually contains detailed information about their chosen mode of delivery, infant feeding choice, client's Viral Load, and CD4 count. Infant postexposure prophylaxis drugs and mother's antiretroviral drugs are given to the women on referral. The women are sent back to the centre at 2 weeks postdelivery with a completed Case Record Form (CRF) designed specifically to capture all delivery-related information. Information on the CRF is used to complete the postnatal data base. The Home-Based Care Team contacts any of the women who did not report back 2 weeks after the expected date of delivery. This is to ascertain the reasons for the default.

### 2.2. Study Design

This is a cross-sectional study that was carried out between 1st September 2009 and 31st November 2009. A semistructured questionnaire was administered to the women who met the inclusion criteria and gave consent to participate in the study. Knowledge of ART was measured by asking some basic questions, which were graded. A score above 70% was classified good while below 70% was not good. Adherence was measured by expressing the number of doses taken as a percentage of the number of doses prescribed. For example if 20 doses are prescribed and 19 doses are taken, adherence is 95% [13].

The article "Pattern and Determinants of Antiretroviral Drug Adherence among Nigerian Pregnant Women" was published in 2012. Journal: J Pregnancy.

### 2.3. Study Population

All pregnant women with known gestational age either by date or early ultrasound seen during the study period and who gave informed consent were enrolled. At the time of the conduct of the study, a total of 273 pregnant HIV-positive women were registered for PMTCT services. The study aimed for a precision of ±5% for a proportion of 50% using 95% confidence interval, therefore, a sample size of 70 subjects was required. In order to increase the power of the study, we decided to enroll all pregnant HIV-positive women who attended PMTCT clinic between 1st September and 31st November 2009 provided the minimum sample size of 70 is met.

### 2.4. Data Management

The enrolled women were interviewed using a semistructured questionnaire containing closed and open-ended questions. The open-ended questions were included to give the women opportunity to freely express themselves without boxing them into closed answers. Information on demographics, socioeconomic characteristics, knowledge of HIV, and antiretroviral drug medication, adherence pattern, reasons for missing drugs, and factors that encourage adherence were also contained in the questionnaire. Data management was with SPSS for windows version 17. The *P* value was based on 95% confidence intervals (CI); a *P* value > 0.05 was not significant (NS).

Descriptive analyses were first performed followed by bivariate analyses of the determinant factors associated with good adherence. The variables that were found significant at this level were added to a multivariate logistic regression model and those with a *P*-value < 0.05 were considered significant in the final multivariate model, calculating odds ratios (OR) and 95% confidence interval (CI).

### 2.5. Ethical Issues

Ethical approval for the study was obtained from the Institutional Review Board, Nigerian Institute of Medical Research, Lagos, Nigeria. Written informed consent was obtained from all women for the use of their data for study however, women who declined consent to participate in study were provided care but excluded from research.

The clinic patients are organized into an independent support group of people living with HIV (Positive Life Organization of Nigeria) that ensures that patients are not stigmatized and discriminated against. This group ensures that no patient is denied requisite care because of failure to participate in any of our studies including this study.

## 3. Results

During the three months study period, one hundred and seventy eligible HIV-positive pregnant women consented and were interviewed. One hundred and thirty seven (80.6%) of the interviewed women reported achieving adherence level of greater or equal to 95% using 3 day recall method, with a nonadherent rate of 19.4%.

The article "Pattern and Determinants of Antiretroviral Drug Adherence among Nigerian Pregnant Women" was published in 2012. Journal: J Pregnancy.

The sociodemographic characteristics of the respondents are shown in Table 1. Majority of the women were aged 30–34 years (52.4%), married (77.1%), have at least one living child (70.0%), employed/working (76.5%), had at least secondary education (81.1%), and from the three major ethnic tribes of Yoruba, Igbo, and Hausa (84.1%).

Pregnancy and HIV-related characteristics are summarized in Table 2. One hundred and forty seven (86.5%) women had disclosed their HIV status and their disclosure was to their partners in most of the cases (97.3%). The majority of the women were on first line HAART regimen (58.2%), while the rest of the women were either on non-HAART prophylactic regimen (24.7%) or 2nd line HAART regimen (17.1%). Only 20.0% and 22.9% of the women have had previous PMTCT experience and were within the first trimester, respectively. Their knowledge of HIV and antiretroviral therapy were very good as over 85% of the respondent had very good knowledge. The use of treatment support was relatively common as greater than half of the women had a treatment supporter (55.9%) who is the husband in 89.5% of the cases.

The outcome of subanalysis of reasons given for adhering to the antiretroviral drugs as prescribed, among the women that had adherence level greater 95%, is shown in Table 3. The desire to ensure that the unborn child is protected from HIV infection was the greatest motivation (51.8%). Some of the written expression of the women, expressing the desire to protect the child as the motivation for adherence includes “*I want to protect my baby,” “I do not want to live with the guilt of infecting my baby,” and “I learnt my baby will not be infected if I take my drugs religiously*.*”* The desire to remain healthy and alive was the other motivator for adhering to the ARV drugs (21.2%). These are some of the respondents' written expression “*I want to live long train my children and fulfill my life dreams,” “To keep me healthy, as I was always on admission in the hospital before I started treatment. I am now okay since I started the ARV drugs.”*

The reasons given by the nonadherent respondents for missing or skipping their drugs are shown in Table 4. Forgetfulness (57.6%), tight work schedule (39.4%), and fear of being identified as HIV positive (63.6%) were the common reasons for skipping or missing drugs among the nonadherent women. The respondents expressed this in written form, for example, “I* get stuck in traffic sometimes on my way home from work and am not comfortable carrying my drugs around or taking them in the public.”*

The article "Pattern and Determinants of Antiretroviral Drug Adherence among Nigerian Pregnant Women" was published in 2012. Journal: J Pregnancy.

Table 5 shows the bivariate analysis of some possible factors associated with good drug adherence. Of the nine variables, only four variables which are marital status (*P* = 0.023), disclosure of HIV status (*P* = 0.000), good knowledge of HIV, and ART (*P* = 0.001 and having a treatment supporter (0.002) were found to be significantly associated with good adherence. However, after subjecting the variables found to be significantly associated with good adherence to multiple logistic regressions while controlling for other potential confounders, only HIV status disclosure (odds ratios: 6.1; CI: 2.8–11.6) and having a treatment partner (odds ratios: 2.5; CI: 1.3–6.7) retained their association with good adherence.

## 4. Discussion

 Effective strategies to reduce mother-to-child transmission of HIV infection are well known and well established [1, 3]. These include the use of ARV drugs, avoiding unplanned and unwanted pregnancy in HIV-positive women, safe delivery and infant feeding options, reduction of unwarranted and unnecessary surgical intervention during pregnancy and labor, prevention of prolonged rupture of membrane, and so forth [1, 3]. Research has also shown that at undetectable viral load, it is possible to achieve zero mother to child transmission of HIV infection [1]. Antiretroviral drugs can only achieve the required effect at adherence level of at least 95% [14]. Poor adherence to antiretroviral drugs has been reported to be the major challenge to achieving the goal of antiretroviral therapy [15]. Many factors have been cited as reasons for nonadherence in HIV-positive adults [10–12, 15–18], but relatively few adherence studies have been done in HIV positive pregnant women [4, 19]. Apart from factors preventing adherence in nonpregnant adults, the nausea and vomiting of pregnancy and possible effect of the drugs on the fetus are additional factors that makes adherence in pregnancy a challenge.

We conducted this study not only to provide this scarce information on adherence in pregnancy but also to generate information that will assist during adherence counseling for pregnant HIV positive women accessing PMTCT services.

The nonadherence rate of 19.4% among our cohort, though comparable to 21.7% reported by Igwegbe et al. in South Eastern Nigeria is much lower than 37.1% and 37.4% reported by Olowookere et al. [10] and Shaahu et al. [11], respectively, from Southwestern Nigeria where present study was conducted. Considering that our study and that of Igwegbe et al. [4] was among pregnant women unlike the two studies by Olowookere et al. [10] and Shaahu et al. [11], it seems that adherence is better in pregnancy. It is not surprising that women are willing and ready to do anything, to ensure the wellbeing of their offspring. The above statement was confirmed in this study in which 51.8% of the adherent women gave the reason of protecting their unborn child from HIV infection as the major motivator for taking their drug as prescribed. The effect of vomiting and nausea of pregnancy was not noticed in this study, as majority of the women are referred patients after HIV diagnosis. At the time, these women present to NIMR HIV treatment centre, the nausea and vomiting of pregnancy would have subsided.

The article "Pattern and Determinants of Antiretroviral Drug Adherence among Nigerian Pregnant Women" was published in 2012. Journal: J Pregnancy.

The free services offered at NIMR, compared to other centres, may have played a great role, as cost of drugs and laboratory services have been shown to be a major barrier to antiretroviral drug adherence [18, 20]. The adherence rate of 99% reported by Jones and Barthlomew [19] among 194 pregnant women where services were completely free gives credence to this assertion. The adherence level of 99% reported above also showed that we need to do a lot of work on issues of adherence. Presently, all patients are counseled prior to the initiation of antiretroviral therapy, but there is need to reevaluate counseling methods and techniques where necessary, aiming to achieve the 99% adherence level reported by Jones and Barthlomew [19].

Encouraging the women to come along with a treatment supporter for the counseling sessions prior to initiation of antiretroviral therapy preferably the partners would help in educating the partners appropriately and improving adherence in the long run.

 Apart from reviewing the counseling techniques, the knowledge of the adherence counselors also needs to be evaluated as their beliefs and attitudes are central to effective counseling.

Among the nonadherent women, similar reasons reported in other studies for missing drugs were found [4, 10, 11, 18]. It, therefore, shows that pregnancy related factors are not the reasons for missing antiretroviral drugs during pregnancy, but as a result of other personal and sociocultural factors. Stigma and discrimination remain an important factor militating against quality HIV care, as 63.6% of women in this study expressed the reason for missing their drugs as afraid of being identified as HIV positive. There is, therefore, the need for continued campaign against stigma and discrimination if we must improve adherence to antiretroviral drugs and uptake of other HIV-related services.

The findings of HIV status disclosure and having a treatment support as factors associated with good adherence after controlling for potential confounders is in agreement with previous studies [8]. With the disclosure of HIV status to partners, who in most cases is the husband, he will not only provide support but will act as treatment partner for the spouse. We, therefore, need to encourage these women, to disclose their status to get the maximal benefit of disclosure. It is important, however, to note that women should not be forced to disclose their status, as HIV status disclosure has been reported to be accompanied by partner violence [21]. Instead women who decline to disclose should be counseled and encouraged until they feel safe to disclose.

The article "Pattern and Determinants of Antiretroviral Drug Adherence among Nigerian Pregnant Women" was published in 2012. Journal: J Pregnancy.

It is important to state that self-report used to measure adherence is not the gold standard for adherence measurement, but it has been reported to be sufficient enough to assess adherence when pill count is not possible and electronic devices and blood ARV blood measurement are not feasible [15].

## 5. Conclusion

In conclusion, this study has shown that good adherence is achievable during pregnancy, however, more has to be done to achieve adherence rate of 99% reported elsewhere. The identified reasons for nonadherence and the effects of status disclosure and having a treatment partner will be used to improve adherence counseling process.

## Figures and Tables

**Table 1:** The sociodemographic characteristics of the women enrolled in the study.

Characteristics	Number of women (%) *N* = 170
Age (years)	
(i) <20	2 (1.2)
(ii) 20–24	20 (11.8)
(iii) 25–29	43 (25.3)
(iv) 30–34	89 (52.4)
(v) 35–39	13 (7.6)
(vi) ≥40	3 (1.8)
Number of living children	
(i) 0	51 (30.0)
(ii) 1–2	67 (39.4)
(iii) >2	52 (30.6)
Marital status	
(i) Married	131 (77.1)
(ii) Not married	39 (22.9)
Occupation	
(i) Housewife	35 (20.6)
(ii) Unemployed	5 (2.9)
(iii) Employed/Working	130 (76.5)
Educational level completed	
(i) No formal education	3 (1.8)
(ii) primary	29 (17.1)
(iii) Secondary	99 (58.2)
(iv) Tertiary	39 (22.9)
Ethnic group	
(i) Yoruba	78 (45.9)
(ii) Igbo	52 (30.6)
(iii) Hausa	13 (7.6)
(iv) Other tribes	27 (15.9)

**Table 2:** The distribution of pregnancy and HIV related characteristics of the women enrolled in the study.

Characteristics	Number of women (%) *N* = 170
HIV status disclosure	
(i) Disclosed	147 (86.5)
(ii) Not disclosed	23 (13.5)
ARV drug regimen	
(i) Mono and Dual therapy	42 (24.7)
(ii) First line HAART	99 (58.2)
(iii) 2nd line HAART	29 (17.1)
Gestational age (weeks)	
(i) Less than 13	39 (22.9)
(ii) 13–28	52 (30.6)
(iii) Greater or equal to 29	79 (46.5)
Previous PMTCT experience	
(i) Yes	34 (20.0)
(ii) No	136 (80.0)
Knowledge of HIV and ART	
(i) Good	146 (85.9)
(ii) Poor	24 (14.1)
Has treatment supporter	
Yes	95 (55.9)
No	75 (44.1)

The article "Pattern and Determinants of Antiretroviral Drug Adherence among Nigerian Pregnant Women" was published in 2012. Journal: J Pregnancy.

**Table 3:** Reason for adherence to ARV drugs among respondents with over 95% drug adherence.

Reason for Adherence	No of respondents (%)*
To protect my unborn child	71 (51.8)
To stay healthy and alive	29 (21.2)
As I was told by counselors	27 (19.7)
Informed by my previous PMTCT experience	16 (11.7)

*No of respondents greater than 137 because of multiple responses.

**Table 4:** Reasons for missing drugs among the 33 respondents that had less than 95% adherence.

Reason for nonadherence	No of respondents (%)*
Forgetfulness	19 (57.6)
Slept off	11 (33.3)
Work schedule	13 (39.4)
Religious activity	9 (27.3)
Food requirement of the drug	7 (21.2)
Afraid of someone identifying my drug as HIV drugs	21 (63.6)

*No of respondents greater than 33 because of multiple responses.

**Table 5:** Factors associated with good adherence among the respondents.

Factors	Adherent respondents (%) *N* = 137	Nonadherent respondents (%) *N* = 33	OR (95% CI)	*P* value
Age (years)				
(i) <20	2 (1.5)	0	1.00	
(ii) 20–35	123 (89.8)	28 (84.9)	1.00	
(iii) ≥35	12 (8.8)	5 (15.1)	2.56 (0.85–7.85)	0.08
Number of living children				
(i) 0	42 (30.7)	9 (27.3)	0.82 (0.28–2.44)	0.88
(ii) 1–2	57 (41.6)	10 (30.3)	1.00	
(iii) >2	38 (27.7)	14 (42.4)	2.10 (0.78–5.75)	0.17
Marital status				
(i) Married	119 (86.9)	12 (36.4)	(1.13–6.79)	0.23
(ii) Not married	18 (13.1)	21 (63.6)	1.00	
Occupation				
(i) Unemployed	28 (20.4)	12 (36.4)	1.00	
(ii) Employed/Working	109 (79.6)	21 (63.6)	0.45 (0.18–1.11)	0.09
Educational level completed				
(i) Less than secondary	26 (19.0)	6 (18.2)	1.00	
(ii) At least Secondary	111 (81.0)	27 (81.8)	1.05 (0.36–3.18)	0.89
HIV status disclosure				
(i) Disclosed	131 (95.6)	16 (48.5)	(3.06–23.6)	0.000
(ii) Not disclosed	6 (4.4)	17 (51.5)	1.00	
Previous PMTCT experience				
(i) Yes	31 (22.6)	3 (9.0)	2.92 (0.78–12.92)	0.13
(ii) No	106 (77.4)	30 (91.0)	1.00	
Knowledge of HIV and ART				
(i) Good	124 (90.5)	22 (66.7)	4.77 (1.73–13.22)	0.001
(ii) Poor	13 (9.5)	11 (33.3)	1.00	
Has treatment supporter				
Yes	85 (62.0)	10 (30.3)	3.76 (1.55–9.26)	0.002
No	52 (38.0)	23 (69.7)	1.00	
